# Assessment of Awareness and Practice toward Diabetic Ketoacidosis among Diabetic Patients and Their Caregivers in Hail Region

This article has been retracted.

**DOI:** 10.1155/2022/2904910

**Published:** 2022-09-28

**Authors:** Nahlah Fahad Alreshidi, Sultan Saud Altamimi, Abdulrhman Naif Alharbi, Fahad Faisal Eid Al-Shamry, Abdulrahman Rabah Alsharari, Abdulrahman Ahmed Alkhateeb, Muhannad Fatim Alharbi

**Affiliations:** College of Medicine, University of Hail, Saudi Arabia

## Abstract

**Introduction:**

Diabetic ketoacidosis (DKA) is one of the most serious consequences of diabetes. This serious issue occurs when the body cannot use the glucose as a source of energy because of a lack in the level of insulin which as consequence will lead to an increased level of glucose resulting in DKA.

**Aim:**

The goal of this study was to increase diabetic patients' and caregivers' awareness and practice of DKA at the community level in Hail City, Saudi Arabia, in 2022. The assessment of people's awareness and knowledge on DKA is importance to support any subsequent actions. *Subjects and Methods*. This is a cross-sectional study conducted in Hail City, Saudi Arabia, among diabetic patients and carers. A self-administered questionnaire in Arabic was given to the target demographic via an internet survey. The questionnaire includes basic demographic data (i.e., age, gender, and marital status), clinical characteristics of the diabetic patients, and a set of questionnaires to assess the awareness and practice of the subjects regarding DKA.

**Results:**

348 surveys were received (51.1% males vs. 48.9% females). A total of 29.9% of patients have been diagnosed with DKA. Out of a possible 14 points, the average awareness score was 5.22 (SD 3.39). Poor awareness levels had been found in nearly 70% of the subjects, 23.6% were moderate, and only 8.6% were considered good. Factors associated with increased awareness were being younger, female gender, unmarried, students, type 1 DM, DKA diagnosis, and having good information about DKA.

**Conclusion:**

The awareness of diabetic patients and their caregivers toward DKA was unsatisfactory. Younger female patients who were single and who had been diagnosed with DKA tend to be more aware of DKA as compared to other subjects. There is a compelling reason to bridge the gaps in the awareness of DKA among the diabetic population and their caregivers in our region.

## 1. Introduction

Nowadays, diabetes mellitus (DM) is considered one of the most important diseases in the world. 300 million people may have DM by 2025 because of comfort living and sedentary lifestyle and increase the incidence of obesity [1]. Diabetes mellitus (DM) is a metabolic disorder characterized by persistently elevated blood sugar levels. DM has greater effect on the metabolism of carbohydrates, lipids, and proteins [2]. Type 1 diabetes (T1DM), type 2 diabetes (T2DM), and gestational diabetes are the three main kinds of diabetes. Type 1 DM usually occurs due to autoimmune destruction of beta cells in the islets of Langerhans in the pancreas, leading to reduction in insulin secretion. Type 2 diabetes, on the other hand, is caused by an impairment in insulin action caused by insulin resistance in body tissues, resulting in a deficiency in glucose entry into body cells [3]. T1DM is considered one of the most common endocrine diseases during childhood and adolescence [4]. Diabetic ketoacidosis is one of the most serious complications of diabetes; this serious issue occurs when the body cannot use the glucose as a source of energy because of lack in the level of insulin which as consequence will lead to increase the level of glucose, and then, the tissue uses the ketone or fatty acid for energy, and diabetic ketoacidosis will occur. Usually DKA is associated with T1DM more often than T2DM; however, DKA can also be seen in the patients with T2DM [5]. The characteristic of DKA is blood glucose > 11 mmol/L, venous pH < 7.3, or bicarbonate < 15 mmol/L and ketonemia with ketonuria [6]. Regarding the risk factors, a study which was conducted in the Al-Baha, Saudi Arabia, shows that positive family history of diabetes is the main risk factor among children with DKA. The same previous study shows that childhood infection is the commonest precipitating factor for the development of DKA in children followed by poor compliance with the insulin therapy [7]. About the symptoms, DKA patients usually presented with polyuria with polydipsia (98%), weight loss (81%), muscles fatigue (62%), dyspnea (57%), vomiting (46%), and preceding illness (40%). These symptoms can damage the respiratory and digestive systems, resulting in respiratory failure and severe abdominal discomfort, which can lead to a coma and death [8]. Many studies worldwide have measured DKA awareness and practice among people with diabetes and their caregivers; few studies have measured in Saudi communities. Therefore, we conducted a cross-sectional online survey to determine baseline awareness of DKA in Hail City. To our knowledge, no previous studies on this topic have been conducted in the Saudi population in Hail City.

## 2. Methodology

348 people from Hail City, Saudi Arabia, participated in this cross-sectional online survey, with a population around 699,774. Based on a confidence interval of 95 percent and an acceptable error margin of 5 percent, the study included basic demographic data (such as age, gender, marital status, education level, occupation, and nationality), clinical features of diabetes patients, and a series of questionnaires to measure the subjects' knowledge and practice of DKA. The Statistical Package for Social Sciences (SPSS) software version 23 was used to analyze all of the data (SPSS Inc., Chicago, IL, USA). Informed consent was required before the online questionnaire could be administered to all participants. The study purpose was explained on an online webpage.

### 2.1. Statistical Analysis

The awareness and practice toward diabetic ketoacidosis among diabetic patients and their caregivers have been assessed by using an 8-item questionnaire, where the correct answers had been identified and were coded with 1 while the incorrect answers had been coded with 0. Question 6 was a multiple response answer with 7 correct answers giving an overall awareness questionnaire of 14 items. The total awareness score has been calculated by adding all 14 items, and a score range from 1 to 14 points has been generated, indicating that the higher the score, the greater the awareness of diabetic ketoacidosis. By using 50% and 75% to determine the level of awareness, patients were classified as having poor awareness if the score was below 50%, 50 to 75% was considered moderate, and above 75% was good awareness toward diabetic ketoacidosis.

Descriptive statistics are summarized as numbers, percentages, mean, and standard deviation. Differences in consciousness scores according to patient sociodemographic characteristics were calculated using the Mann–Whitney *Z*-test and the Kruskal-Wallis *H*-test. Normality tests were performed using the Shapiro-Wilk test and the Kolmogorov-Smirnov test. Consciousness scores are considered anomalous distributions. Thus, nonparametric tests were applied. A *P* value of 0.05 was considered statistically significant. The data were analyzed using Statistical Packages for Social Sciences (SPSS) version 26 (Armonk, NY: IBM Corp, USA).

## 3. Results

There were 348 surveys received in total. The sociodemographic characteristics of the respondents are detailed in Table 1. 51.1 percent were over 35 years old, with males accounting for more than half (51.1%) and Saudis accounting for nearly all (96.6%). Respondents who were married constituted 62.6%, and those with university degree holders were 61.5%. With respect to occupation, half of them (50%) were employed.

Table 2 shows that 76.4 percent of patients had been diagnosed with diabetes, with type 2 diabetes being the most common kind (40.2 percent). Of them, diabetes duration between 1 and 5 years was reported by 47.7% of the patients. A total of 29.9% of patients have been diagnosed with DKA. In addition, 93.1% believed that there was a lack of education for DM patients about DKA in Hail City.

Regarding Figure 1, the most commonly known source for DKA information was a doctor (27.6%), followed by the Internet (17.2%), and family and friends (14.9%).

The assessment of awareness toward DKA is given in Table 3. It can be observed that 43.7% of the respondents were correct that DKA is considered to be an emergency complication of DM that required urgent intervention. Only 17.8% of the respondents were aware that DKA is not only for children. Approximately one quarter (25.3%) of the subjects knew that one of the main causes of DKA was the lack of insulin in the blood which may be related to forgetting to take insulin injections. More than half (51.1%) believed that maintaining the normal level of A1c reduces the incidence of DKA. 40.8% indicated that for an incidence of DKA, the most common action to be taken was to call an ambulance and bring the patient to the hospital immediately. The most common symptoms of DKA were feeling exhausted/fatigued (64.9%), followed by nausea (48.9%) and unconsciousness (45.4%). Only 27% and 24.7% of the respondents knew that infection and physical exertion can cause DKA. The overall mean awareness score was 5.22 (SD 3.39) based on the preceding assertions, with poor, moderate, and good awareness level finding in 67.8%, 23.6 percent, and 8.6 percent, respectively (Figure 2).

When the disparities in awareness scores were compared to the sociodemographic features of participants, it was shown that a greater awareness score was more closely related with those who were younger in age (*Z* = 3.724; *P* < 0.001), gender female (*Z* = 3.218; *P* = 0.001), being unmarried (*Z* = 2.631; *P* = 0.009), being a student (*H* = 34.961; *P* < 0.001), having type 1 diabetes (*Z* = 4.938; *P* < 0.001), DKA diagnosis (*Z* = 7.076; *P* < 0.001), and having good information about DKA (*Z* = 12.040; *P* < 0.001) while the differences in the score of awareness according to education, respondents with DM, duration of DM, and opinion that there was a lack of DKA education in Hail City did not reach statistical significance (*P* > 0.05) (Table 4).

## 4. Discussion

The goal of this study is to find out how well diabetic patients and their carers understand and practice diabetic ketoacidosis. The results of this study showed that there was a lack of awareness of DKA among our sample population. More than two-thirds (67.8%) of the subjects were assumed to have poor awareness levels, 23.6% were moderate, and only 8.6% were good (mean score: 5.22; SD 3.39, out of 14 total score points). Consistent with our findings, Alanazi et al. [5] reported that more than half (54%) of the diabetic patients in Riyadh City, Saudi Arabia, demonstrated low knowledge about the risk factors of DKA. Our reports were likewise in line with Satti et al.'s publication [8]. According to their accounts, insufficient awareness was detected among patients regarding the risk factors, complications, and management of DKA while in India [9, 10], and most diabetic patients (80%) appeared to have a poor level of DKA knowledge. However, in a study published in Somalia [11–13], the knowledge, attitude, and practice of the patients who visited Egyptian Hospital in Mogadishu, Somalia, regarding diabetic complications were satisfactory which was better than our reports. The current gap in awareness may not only sustain a significant burden with the cost of treatment on the patients and their families but it may also lead to severe complications that can be life-threatening if not diagnosed and treated early. Thus, health education among these groups of patients is imperative.

Younger female patients who were unmarried and currently studying were more associated with having better awareness levels, but the differences in the awareness levels between the more educated subjects and less educated ones did not reach statistical significance (*P* = 0.057). In a study conducted in India [10, 14], they found a significant relationship between educational status and the knowledge about DKA while in Abha, Saudi Arabia [12, 13, 15, 16], low knowledge levels were more common among less-educated parents, being a father aged more than 40 years, unemployed or those nonhealthcare parents, and having a lower monthly income which contradicted our reports. Furthermore, we observed that patients who have been diagnosed with type 1 DM with associated DKA were seen to have an increased level of awareness. In addition, our results also suggested that respondents who had good information about DKA were likely to have a better understanding of the complications of diabetes. The factors associated with awareness level are necessary to identify as this can guide patients in the management of their disease. As a result, further research is needed to determine the factors that influence diabetes patients' understanding of risk factors, consequences, and prevention of DKA.

In a study published by Satti et al. [4], they discovered that infections were the major cause of DKA (82.1%), and the most common presenting symptoms were vomiting (71.3%) and stomach pain (66.3 percent). In another report published in the Central region, KSA [16], the scent of breathing was the most well-known symptom of DKA (70 percent), whereas skin coldness was the least well-known (29.5 percent). In addition, the author found out that 68.8% were aware that DKA could lead to coma or severe dehydration (63.3%). However, in our study, only 27% of our sample was aware that infection can cause DKA and only 24.7% knew that physical exertion can also lead to DKA. On the other hand, we noted that our population believed that tiredness and exhaustion (64.9%) were the major presenting symptoms of the disease.

Only 43.7% of our sample population believed that DKA was an emergency complication of DM which requires immediate treatment. However, suboptimal awareness accounts for whether DKA can only affect children and what complications might occur for the lack of insulin in the blood was suboptimal. Despite these shortcomings, some of our population rely on their information by visiting a doctor (29.9%), the Internet (17.2%), and family and friends (14.9%). Among diabetic patients in Somalia [11], 37.5% of them visited a doctor to get advice regarding issues about their disease and their adherence to regular exercise was also low which may result in more complications of the disease.

In a study done in Riyadh, KSA [17, 18], 68.8% of diabetic caregivers were sure that DKA could lead to coma or severe dehydration (63.3%) with 88.9% who knew that DKA can be prevented by taking insulin as instructed. In our study, only a quarter (40.8%) were confident that for an incidence of DKA, the most important action to be taken was to rush the patient to the hospital to get immediate treatment; however, only 25.3% of our sample was aware that neglecting insulin shot could lead to DKA. Diabetes educators should instruct patients and caregivers that for any signs of DKA, insulin administration should never stop, and they must do self-monitoring of blood glucose and increase the dose if needed. Hence, they must go to the emergency room to prevent further complications of DKA if all options failed to improve the patient.

## 5. Conclusion

The awareness of diabetic patients and their caregivers toward DKA was unsatisfactory. Younger female patients who were single and who had been diagnosed with DKA tend to be more aware of DKA as compared to other subjects. There is a compelling reason to bridge the gaps in the awareness of DKA among the diabetic population and their caregivers. Collective efforts are important to educate our diabetic patients as well as their caregivers regarding the risk factors and complications of diabetes. Also, it is worthwhile to raise their awareness about the most important symptoms of DKA and the immediate action to be done for any incidence of this type of diabetes complication. Further research is warranted in order to establish the awareness and practice levels of diabetic patients along with their caregivers in our region.

## Figures and Tables

**Figure 1:** Sources of information regarding DKA.

**Figure 2:** Level of awareness toward DKA.

**Table 1:** Sociodemographic characteristics of the diabetic patients (*n* = 348).

Study variables	*N* (%)
Age group	
(i) 18–20 years	42 (12.1%)
(ii) 21–25 years	58 (16.7%)
(iii) 26–30 years	34 (09.8%)
(iv) 31–35 years	36 (10.3%)
(v) >35 years	178 (51.1%)
Gender	
(i) Male	178 (51.1%)
(ii) Female	170 (48.9%)
Nationality	
(i) Saudi	336 (96.6%)
(ii) Non-Saudi	12 (03.4%)
Marital status	
(i) Single	114 (32.8%)
(ii) Married	218 (62.6%)
(iii) Divorced	16 (04.6%)
Educational level	
(i) Primary or below	32 (09.2%)
(ii) Elementary	26 (07.5%)
(iii) High school	76 (21.8%)
(iv) University	214 (61.5%)
Occupation	
(i) Student	72 (20.7%)
(ii) Employed	174 (50.0%)
(iii) Unemployed	102 (29.3%)

**Table 2:** Clinical characteristics of the diabetic patients (*n* = 348).

Variables	*N* (%)
Diagnosed with diabetes	
(i) Yes	266 (76.4%)
(ii) My son/daughter has diabetes	82 (23.6%)
Type of diabetes	
(i) Type 1	136 (39.1%)
(ii) Type 2	140 (40.2%)
(iii) I do not know	72 (20.7%)
Duration of diabetes	
(i) Between 1 and 5 years	166 (47.7%)
(ii) Between 6 and 10 years	94 (27.0%)
(iii) More than 10 years	88 (25.3%)
Diagnosed with DKA	
(i) Yes	104 (29.9%)
(ii) No	244 (70.1%)
Having good information about DKA	
(i) Yes	104 (29.9%)
(ii) No	244 (70.1%)
In your opinion, is there a lack of education for diabetic patients about diabetic ketoacidosis in Hail City?	
(i) Yes	324 (93.1%)
(ii) No	24 (06.9%)

**Table 3:** Assessment of awareness toward diabetic ketoacidosis among the diabetic patients (*n* = 348).

Awareness statement	*N* (%)
(1) Diabetic ketoacidosis is considered to be as follows:	
(i) An emergency complication of diabetes that requires urgent treatment^∗^	152 (43.7%)
(ii) One of the chronic complications of diabetes and does not require a visit to a doctor; it can be treated at home	24 (06.9%)
(iii) I do not know	172 (49.4%)
(2) Diabetic ketosis only affects children	
(i) Yes	58 (16.7%)
(ii) No^∗^	62 (17.8%)
(iii) I do not know	228 (65.5%)
(3) One of the main causes of diabetic ketoacidosis	
(i) Lack of insulin in the blood due to forgetting to take insulin injections^∗^	88 (25.3%)
(ii) High blood sugar due to irregular eating and exercise	100 (28.7%)
(iii) I do not know	160 (46.0%)
(4) Maintaining the normal level of A1c reduces the incidence of diabetic ketoacidosis	
(i) Yes^∗^	178 (51.1%)
(ii) No	20 (05.7%)
(iii) I do not know	150 (43.1%)
(5) If a diabetic patient suffers from diabetic ketoacidosis, the treatment is as follows:	
(i) Give the patient oral sugar, and wait until they get better	44 (12.6%)
(ii) Call an ambulance, and take him to the hospital immediately^∗^	142 (40.8%)
(iii) I do not know	162 (46.6%)
(6) The most important symptoms that indicate that a diabetic patient has diabetic ketoacidosis^†^	
(i) Feeling tired and exhausted/fatigue^∗^	226 (64.9%)
(ii) Nausea^∗^	170 (48.9%)
(iii) Unconsciousness^∗^	158 (45.4%)
(iv) Stomach ache^∗^	128 (36.8%)
(v) Difficulty breathing or rapid breathing^∗^	126 (36.2%)
(vi) Distinctive breath smell^∗^	112 (32.2%)
(vii) Blurred vision^∗^	94 (27.0%)
(7) Infection (bacterial, viral, or fungal) may be a cause of diabetic ketoacidosis?	
(i) Yes^∗^	94 (27.0%)
(ii) No	68 (19.5%)
(iii) I do not know	186 (53.4%)
(8) Physical exertion may be a cause of diabetic ketoacidosis?	
(i) Yes^∗^	86 (24.7%)
(ii) No	108 (31.0%)
(iii) I do not know	154 (44.3%)
Awareness score (mean ± SD)	5.22 ± 3.39
Level of awareness	
(i) Poor	236 (67.8%)
(ii) Moderate	82 (23.6%)
(iii) Good	30 (08.6%)

∗ indicates correct answer. ^†^Variable with multiple response answers.

**Table 4:** Differences in the score of awareness according to the sociodemographic characteristics of the diabetic patients (*n* = 348).

Factor	Awareness score (14) Mean ± SD	*Z*/*H*-test	*P* value
Age group^a^			
(i) ≤35 years	5.85 ± 3.38	*Z* = 3.724	<0.001^∗∗^
(ii) >35 years	4.62 ± 3.29		
Gender^a^			
(i) Male	4.73 ± 3.44	*Z* = 3.218	0.001^∗∗^
(ii) Female	5.73 ± 3.26		
Marital status^a^			
(i) Unmarried	5.82 ± 3.48	*Z* = 2.631	0.009^∗∗^
(ii) Married	4.86 ± 3.29		
Educational level^a^			
(i) High school or below	5.49 ± 3.06	*Z* = 1.906	0.057
(ii) University	5.05 ± 3.58		
Occupation^b^			
(i) Student	7.00 ± 3.46	*H* = 34.961	<0.001^∗∗^
(ii) Employed	4.28 ± 2.99		
(iii) Unemployed	5.57 ± 3.43		
Diagnosed with diabetes^a^			
(i) Yes	5.23 ± 3.53	*Z* = 0.394	0.693
(ii) My son/daughter has diabetes	5.19 ± 2.89		
Type of diabetes^a^			
(i) Type 1	6.51 ± 3.42	*Z* = 4.938	<0.001^∗∗^
(ii) Type 2	4.56 ± 3.38		
Duration of diabetes^b^			
(i) Between 1 and 5 years	5.19 ± 2.89	*H* = 2.343	0.310
(ii) Between 6 and 10 years	5.53 ± 3.80		
(iii) More than 10 years	4.93 ± 3.79		
Diagnosed with DKA^a^			
(i) Yes	7.09 ± 3.15	*Z* = 7.076	<0.001^∗∗^
(ii) No	4.42 ± 3.17		
Having good information about DKA^a^			
(i) Yes	8.69 ± 2.85	*Z* = 12.040	<0.001^∗∗^
(ii) No	3.74 ± 2.37		
In your opinion, is there a lack of education for the diabetic patients about diabetic ketoacidosis in Hail City?^a^			
(i) Yes	5.19 ± 3.35	0.499	0.618
(ii) No	5.67 ± 3.94		

^a^The Mann–Whitney *Z*-test was used to get the *P* value. ^b^The Kruskal Wallis *H*-test was used to get the *P* value. ^∗∗^At the 0.05 level, the difference is significant.

## Data Availability

The data used to support the findings of this study are included within the article.
